# TRIM proteins in neuroblastoma

**DOI:** 10.1042/BSR20192050

**Published:** 2019-12-23

**Authors:** Yonghu Xu, Zihan Zhang, Guofeng Xu

**Affiliations:** Department of Pediatric Urology, Xinhua Hospital, National Key Clinical Specialty, Shanghai Top-Priority Clinical Center, School of Medicine, Shanghai Jiaotong University, Shanghai 200092, China

**Keywords:** E3 ubiquitin ligase, neuroblastoma, TRIM proteins, ubiquitination

## Abstract

Neuroblastoma (NB) is the most common extracranial solid tumor in childhood. Outcome for children with high-risk NB remains unsatisfactory. Accumulating evidence suggests that tripartite motif (TRIM) family proteins express diversely in various human cancers and act as regulators of oncoproteins or tumor suppressor proteins. This review summarizes the TRIM proteins involving in NB and the underlying molecular mechanisms. We expect these new insights will provide important implications for the treatment of NB by targeting TRIM proteins.

## Introduction

Neuroblastoma (NB) is the most common extracranial solid tumor in childhood, accounting for 8–10% of all children’s malignancies and about 15% of cancer-related deaths [1,2]. NB onset has a strong genetic component, with gene mutations commonly seen in MYCN, ALK and PHOX2B [3]. In addition, clinical outcomes of NB patients are highly heterogeneous, with differentiation status [4], disease stage [5], age at diagnosis [6] and MYCN amplification [7] all influencing prognosis. What’s more, genome sequencing studies revealed that the genetic variations of NB tumor are markedly lower than that found in many other adult solid tumors [8], indicating the importance of post-translational modification in the occurrence and development of NB. As a vital post-translational modification, ubiquitination is involved in the regulation of many eukaryotic signaling pathways and aberrant ubiquitin signaling is currently an active area in NB research. For example, recent studies have indicated ubiquitination modification functions as an important regulator for the stability of MYCN protein, a marker of poor NB prognosis [9]. Ubiquitin-specific protease 7 (USP7) promotes the growth of MYCN-amplified NB cell lines by inducing the deubiquitination and subsequent stabilization of MYCN [10], while the ubiquitin-ligase FBW7 promotes the proteasome-mediated MYCN degradation and leads to the opposite result [11].

The tripartite motif (TRIM) family proteins, also known as RBBC proteins, are characterized by the common presence of RBBC motif comprises a RING domain, either one or two B-boxes (B1 and B2), and a coiled-coil (CC) domain in their amino terminal, followed by a highly variable carboxyl-terminal domain, which categorizes them into 11 subgroups (C-I – C-XI, Figure 1) [12,13]. In recent years, accumulating studies have found that TRIM proteins regulate a wide variety of biological processes and their dysregulation are associated with various diseases, including cancer [14–16]. The functions of TRIM proteins in tumor development and progression are complex and diverse. There are several established mechanisms of carcinogenesis involving the TRIM family, including: (1) Acquiring oncogenic potential through chromosomal translocations. One best-known example is TRIM19, which is encoded by the promyelocytic leukaemia (PML) gene and involves in the balanced translocation with retinoic acid receptor-α (RARα) to produce the PML-RARα fusion protein. This kind of fusion protein specifically occurs in patients with acute promyelocytic leukaemia (APL) [17], acting as a RARα transcriptional suppressor and thus inducing a block in the differentiation of promyelocytes, which is the underlying etiology of this blood cancer [18,19]. (2) Regulating the activation of nuclear receptors, such as androgen receptors (AR) and estrogen receptors (ER). For example, both TRIM24 and TRIM68 can interact with the AR and increase its transcriptional activity in the presence of dihydrotestosterone (DHT) in prostate cancer cells [20,21]. Several findings also indicate that TRIM proteins regulate transcription by modifying chromatin. For instance, TRIM16 has been shown to increase histone acetylation and reactivate the transcription of retinoic acid receptor β2 (RARβ2) in retinoid-resistant breast and lung cancer cells [22]. (3) Functioning as E3 ubiquitin ligases to regulate the degradation of oncoproteins and tumor suppressor proteins. For example, TRIM11 exerts its oncogenic effect in hepatocellular carcinoma through the inhibition of p53 [23], while TRIM67 suppresses colorectal cancer initiation and progression via the activation of p53 [24]. TRIM65 enhances the invasiveness of bladder urothelial carcinoma (BUC) cells by inducing epithelial–mesenchymal transition (EMT) and promoting the ubiquitination and degradation of Annexin A2 (ANXA2) [25].

**Figure 1:** TRIM proteins domain structure and classification of TRIMs (C-I to C-XI) TRIMs have an N-terminal RING finger (R), one or two B-boxes (B1 and B2), and coiled coil (CC) domain. C-terminal domains comprise various domains including: ARF, ADP-ribosylation factor family domain; BROMO, bromodomain; COS, cos-box; FIL, filamin-type Ig domain; FN3, fibronectin type III repeat; MATH, meprin and TRAF-homology domain; NHL, NCL1, HT2A and LIN41 domain; PHD, PHD domain; PRY, PRY domain; SPRY, SPRY domain; TM, transmembrane region. Dashed-outline domains are those which are differentially present among subfamily members.

The involvement of TRIM protein family in various oncogenic processes makes it a current focus in cancer research. While the functions of TRIM proteins in multiple cancers have been described, their roles in NB have only recently begun to emerge and poorly understood. In this review, we summarize the current research progress of TRIM proteins in NB (Table 1).

**Table 1:** TRIM proteins and their roles in regulating neuroblastoma

TRIM proteins	Functions	References
TRIM11	Interacting with PHOX2B and increasing the expression of DBH	[33]
TRIM16	Enhancing retinoic acid receptor β (RAR-β) transcription	[23,43]
	Down-regulating cytoplasmic vimentin and nuclear E2F1	[45]
	Regulating G1/S cell cycle progression	[46]
	Modulating activity of caspase-2 and promoting apoptosis	[47]
TRIM17	Repressing apoptosis by stabilizing anti-apoptotic proteins Mcl-1	[51,52]
TRIM32	Enhancing transcriptional activity of RARα	[63]
	Inducing asymmetric cell division (ACD)	[64]
	Facilitating c-MYC and n-MYC proteasomal degradation	[62,64]
TRIM36	Being hypermethylated in neuroblastoma tumors	[72]
TRIM59	Inducing the expression of ANXA2	[78]
	Regulating Wnt/β-catenin signaling pathway	[80]

## TRIM11

TRIM11, also known as ring finger protein 92 (RNF92), belongs to the C-IV subfamily, containing a RING finger, one B-box domain, a coiled-coil domain and a C-terminal PRY domain and SPRY domain. As an E3 ubiquitin ligase, it is reported to be up-regulated in several human tumors. In lung cancer, TRIM11 is up-regulated and correlates with poor prognosis [26]. In lung adenocarcinoma, TRIM11 promotes tumor angiogenesis through activating transcription 3 (STAT3)/vascular endothelial growth factor A (VEGFA) pathway [27]. In hepatocellular carcinoma (HCC), enforced expression of TRIM11 promotes cell proliferation, invasion, and migration by activating of the PI3K/Akt signaling pathway [28]. A recent study also revealed that TRIM11 regulates the proliferation and apoptosis of breast cancer cells by regulating ERK1/2 and JNK1/2 signaling pathways [29]. These results indicate that TRIM11 is responsible for different oncogenic processes in various cancers.

Of interest, TRIM11 has recently been shown to involve in the process of neurogenesis. For example, it has been shown to mediate the degradation of PAX6 (a member of the paired-box family of transcription factors which play key roles in development) via the ubiquitin–proteasome system, thereby modulating cortical neurogenesis [30]. TRIM11 has also been reported to be strongly correlated with the differentiation status of malignant glioma cells [31]. More interestingly, TRIM11 can interact with Paired-Like Homeobox 2B (PHOX2B), a homeodomain transcription factor [32], to increase the expression of dopamine β hydroxylase (DBH) gene and participate in the development of noradrenergic (NA) neurons [32].

Universally known, NB originates from sympathoadrenal precursor cells of the sympathetic nervous system and the tumor cells have embryonic features, presumably as a consequence of an impaired capacity to respond to signals operating during normal differentiation [33]. Moreover, PHOX2B, whose coding gene is located on chromosome 4p13, is originally found in a NB cell line. It is expressed specifically in the nervous system and has a vital effect on the formation and differentiation of sympathetic neurons and chromaffin cells [34]. In addition, it has been reported that PHOX2B germline mutations, which account for 6% hereditary NBs, are involved in the initiation of NB tumorigenesis [35]. Thus, these findings provide the potential role of TRIM11 in NB by regulating PHOX2B.

## TRIM16

TRIM16, also named as the estrogen responsive B box protein (EBBP), has been shown to play a negative role in the development and progression of several cancers. For example, the expression of TRIM16 is significantly down-regulated in HCC and knockdown of TRIM16 enhances HCC cell migration and invasion via the promotion of EMT process [36]. TRIM16 is also at low levels in prostate tumors and enforced expression of TRIM16 inhibits prostate cancer cell migration and invasion in a manner associated with the inhibition of Snail signaling pathway and EMT process [37]. The anti-tumor function of TRIM16 has also been elucidated in many other cancers, such as ovarian cancer [38], breast cancer [39], non-small cell lung cancer [40] and melanoma [41]. Together, these studies indicate a tumor-suppressing function for TRIM16 in human cancers.

Recent studies have demonstrated that TRIM16 acts as a tumor suppressor in NB. First, TRIM16 can enhance the transcription of retinoic acid receptor β (RARβ), and overexpression of TRIM16 significantly reduces the proliferation of RA-sensitive NB cells as well as RA-resistant lung and breast cancer cells [42]. These findings suggest an important role of TRIM16 in the response of these tumor cells to differentiating agents, such as RA, an effective inducer of NB cell differentiation that has been used in the clinic for the treatment of high-risk NB [43]. Further investigation showed that TRIM16 can reactivate the transcription of RARβ2 by increasing histone H3 acetylation, with the de-acetylation of histone H3 considered to be the most common mechanism of RARβ2 transcriptional repression in retinoid-resistant cancer cells [22]. These studies suggest that TRIM16 may modulate the transcriptional activity of RA-related receptors that required for NB cell differentiation and could be a novel therapeutic target for retinoid-resistant NB cancer. Second, TRIM16 can affect the migration and differentiation of NB cell through down-regulating vimentin and nuclear E2F1 protein (required for cell replication) [44]. TRIM16 can also influence NB proliferation *in vitro* and tumorigenicity *in vivo* through the regulation of cell cycle [45]. Third, TRIM16 can promote the apoptosis of BE(2)-C NB cells by directly interacting with caspase-2 and modulating its activity [46]. In conclusion, results above have suggested that TRIM16 serves as a tumor suppressor in NB, and defining an effective method to increase TRIM16 protein expression in NB might provide a novel strategy of the cancer therapy.

## TRIM17

TRIM17, also known as Testis RING finger protein (TERF), is expressed not only in the testis but also in the brain during embryonic development [12], suggesting it may have a role in neuronal development. In a previous study, TRIM17 has been identified as a crucial E3 ubiquitin ligase that is necessary for neuronal apoptosis [47]. Unlike majority of TRIM proteins, such as TRIM5α, TRIM6, TRIM20 and TRIM21, which have been demonstrated to promote autophagy, TRIM17 is notable because it can inhibit autophagy [48]. Since neuronal apoptosis is crucial for normal development of the nervous system [49] and NB originates from precursor cells of the sympathetic nervous system, this suggests that TRIM17 may has some effects on NB.

Indeed, several studies *in vivo* in NB cells have shown the function of TRIM17 in promoting neuronal apoptosis. For instance, in NB Neuro2A cells, TRIM17 mediates the ubiquitination and degradation of Mcl-1, an anti-apoptotic Bcl-2 family protein that is necessary for initiating neuronal apoptosis [50]. TRIM17 has also been reported to stabilize BCL2A1, another anti-apoptotic Bcl-2 family protein that contributes to chemo-resistance in a subset of tumors [51]. In summary, these results suggest that TRIM17 is an important factor in neuronal apoptosis. However, studies on the function of TRIM17 in human cancers are still lacking. Whether the function of TRIM17 contributes to NB tumor onset and progression is not yet clear.

## TRIM32

TRIM32 is known as Limb Girdle Muscular Dystrophy 2H (LGMD2H), based on the finding that TRIM32 deficiency in mice results in phenotypes characteristic of the human disease [52]. A role for TRIM32 in the regulation of skeletal muscle stem cell differentiation and normal adult muscle regeneration has been reported [53]. Moreover, TRIM32 is reported to exhibit tumor suppressor functions in many human cancers, including breast cancer, gastric cancer, lung cancer and skin cancer [54–57]. Mechanistically, TRIM32 is an E3 ubiquitin-ligase for some tumor suppressors, such as p53 and Abi2 (Abl-interactor 2) and can regulate their degradation [58,59]. In addition, TRIM32 can promote the proliferation and invasion of gastric cancer cell lines by activating β-catenin signaling pathway [55]. All these findings suggest that TRIM32 is involved in tumor formation and development.

Previously, several studies have shown the importance of TRIM32 in neuronal differentiation by several different mechanism as follows: First, TRIM32 can ubiquitylate and result in the proteasomal degradation of c-Myc, one of the key stem cell transcription factors (SCTFs) crucial for neuronal stem cell (NSC) renewal and maintaining an undifferentiated phenotype [60,61]. Second, TRIM32 can interact with RARα and enhance its transcriptional activity, bringing about enhancement of neural differentiation [62]. These findings suggest that TRIM32 may play an important role in the process of neural differentiation and can be a tumor-suppressor candidate of NB. Indeed, TRIM32 concentrates in one of the daughter cells during mitosis, where it interacts with MYCN and facilitates its proteasomal degradation, thus inducing asymmetric cell division (ACD) of human NB cells, resulting in one cell with neural progenitor cell activity and the other with potential for differentiation [63]. Furthermore, N-myc downstream regulated gene 2 (NDRG2), a new tumor suppressor gene that has recently been reported to suppress the growth and aggressiveness of NB cells [64], is identified as a novel target for TRIM32 [65]. Together, the above-mentioned studies provide some support for us to consider TRIM32 as a tumor suppressor in NB, offering an alternative direction for NB prognosis and/or treatment.

## TRIM36

TRIM36, also known as ring finger protein 98 (RNF98), belongs to the C-I subfamily and contains a RING finger, one B-box domain, a coiled-coil domain and C-terminal domains (COS domain, FN3 domain and PYR domain). It is located in the tumor suppressor gene region at chromosome 5q22.3 [66], and has been reported to be an E3 ubiquitin-ligase for p53, one of the best-known tumor suppressors [67]. Overexpression of TRIM36 decelerates the cell cycle and limits cell growth [68]. TRIM36 can also act as a putative tumor suppressor by attenuating MAPK/ERK signaling pathways and regulating apoptosis-related pathways in prostate cancer [69,70]. These findings indicate that TRIM36 may have suppressive effects on tumors, specifically in prostate cancer.

In agreement with above hypothesis, genome-wide methylation analysis on 60 NB tumors using Illumina 450K methylation arrays revealed that TRIM36 is hypermethylated and has lower expression in aggressive NB tumors compared with less aggressive ones [71], indicating that down-regulated TRIM36 has a significant correlation with NB tumor pathogenesis and progression. Furthermore, there is an observed trend for better survival in NB patients with high TRIM36 expression indicated by bioinformatic analysis of public available Kocak datasets, which were obtained from the R2 Genomics Analysis and Visualization Platform (http://r2.amc.nl) (Figure 2). The same trend is seen in other NB datasets, such as SEQC and Oberthuer. The data presented above suggests that TRIM36 probably plays a negative role in NB development and progression. Unfortunately, information in regards to the specific roles of TRIM36 in NB is currently limited, and additional research is required in this area.

**Figure 2:** Kaplan–Meier analysis of overall survival (left side) and event-free survival (right side) for the Kocak datasets based on TRIM36 expression with the log-rank test *P* value indicated (*n* = 649, with 173 samples lack survival data and being omitted from the analysis)

## TRIM59

TRIM59, also known as mouse ring finger protein 1 (MRF1), belongs to the C-XI TRIM subfamily with a RING finger, one B-box domain, a coiled-coil domain and a C-terminal trans-membrane region [72]. TRIM59 is found, among all the TRIM genes, to be the only member displaying marked up-regulation across all 12 cancer types in The Cancer Genome Atlas (TCGA) database [73], suggesting a probably oncogenic function of it in human cancers. Indeed, there is expanding evidence that TRIM59 is an important regulator of tumorigenesis. For instance, TRIM59 is highly expressed and acts as an early signal transducer of Ras signaling pathway in prostate cancer (CaP) mouse models, whereas the silencing of TRIM59 results in inhibition of cell growth and S-phase arrest in CaP cells [74]. Immunohistochemical analysis shows that TRIM59 expression is significantly up-regulated in multiple human cancers and overexpressed TRIM59 is associated with tumorigenesis and progression [75]. A study in glioblastoma (GBM) cells suggests that TRIM59 promotes GBM tumorigenesis through interaction with nuclear STAT3 and maintains its transcriptional activation by preventing its dephosphorylation [76].

Intriguingly, TRIM59 can induce the expression of ANXA2 [77], a protein that has been reported to enhance multidrug resistance in NB from work in my laboratory [78]. More interestingly, TRIM59 knockdown inhibits cell proliferation by downregulating the Wnt/β-catenin signaling pathway in human NB cells [79]. Collectively, these data imply a role of TRIM59 in NB progression. However, there is currently limited study on the role of TRIM59 in NB. Thus, further investigations are needed to understand its precise function and importance in this pediatric cancer.

## Conclusion and perspectives

As an important post-translational modification, ubiquitination has received much attention for its wide and complex roles in many cellular processes, including protein degradation, cell survival and differentiation, innate and adaptive immunity, and signal transduction [80]. In particular, there has been some success in the use of drugs that act on ubiquitination pathway, such as proteasome inhibitors bortezomib and carfilzomib, which are approved by US FDA to be used for the treatment of multiple myeloma [81]. In parallel, targeting E3 ligases or deubiquitinating enzymes has also been a research focus in anti-tumor drug discovery. For example, the successful use of arsenic trioxide (ATO) to treat APL with PML (TRIM19)–RARα fusion protein. Compared with bortezomib treatment, which often leads to multiple side effects and drug resistance, drugs that specifically target E3 ubiquitin ligases, are likely to be more effective in the treatment of of different cancers due to their high substrate specificity. TRIM proteins, the largest subfamily of RING E3 ligases, are potentially strong candidates for therapeutic targeting as they are reported to be associated with cancer by mechanism including involvement in p53 pathway, activation of nuclear receptors and regulation of oncoproteins and tumor suppressors with their E3 ligase activity [16].

As noted above, recent genome sequencing studies revealed relatively low level of gene mutations in NB, suggesting that epigenetic regulation of gene expression may play an important role in the occurrence and development of NB. Thus, there are substantial biomedical research focusing on the contributions of post-translation modification to the origin and progression of NB. As we have discussed in this review, there are six TRIM proteins known to positively or negatively regulate the initiation or progression of NB, suggesting these TRIM proteins would be attractive drug targets for the disease. However, other TRIM proteins which are known to involve in tumorgenesis but not studied explicitly in NB, may play roles in the development of NB as well, such as TRIM protein regulating nuclear receptors (including TRIM19, TRIM24, TRIM25 and TRIM68) and the p53 pathway (including TRIM13, TRIM19, TRIM24, TRIM28 and TRIM29). Moreover, while other TRIM proteins are associated with the prognosis of some cancers, including NB, their precise mechanisms of action and contributions to cancer remain largely unknown. In addition, there are no current drugs targeting TRIM proteins at the laboratory or clinical level for tumor therapy. Thus, further detailed analysis of TRIM proteins is important to understand how to control TRIM proteins as seeds for effective therapy of NB in aim to improve the curative effect and prognosis of the disease.

## Abbreviations

ACD: asymmetric cell division
ANXA2: Annexin A2
APL: acute promyelocytic leukaemia
AR: androgen receptor
ATO: arsenic trioxide
BUC: bladder urothelial carcinoma
CaP: prostate cancer
DBH: dopamine β hydroxylase
DHT: dihydrotestosterone
EBBP: estrogen responsive B box protein
EMT: epithelial–mesenchymal transition
ER: estrogen receptor
GBM: glioblastoma
HCC: hepatocellular carcinoma
LGMD2H: limb girdle muscular dystrophy 2H
MRF1: ring finger protein 1
NB: neuroblastoma
NDRG2: N-myc downstream regulated gene 2
NSC: neuronal stem cell
PHOX2B: paired-like homebox 2B
PML: promyelocytic leukaemia
RARα: retinoic acid receptor-α
RARβ2: retinoic acid receptor β2
RNF92: ring finger protein 92
RNF98: ring finger protein 98
SCTF: stem cell transcription factor
TERF: testis RING finger protein
TRIM: tripartite motif
USP7: ubiquitin-specific protease 7
